# Prevention of Business Risks of Internet Information Security Platforms Based on Blockchain Technology

This article has been retracted.

**DOI:** 10.1155/2022/7671810

**Published:** 2022-03-15

**Authors:** Bingqing Yang

**Affiliations:** College of Information Engineering, Fuyang Normal University, Fuyang 236041, Anhui, China

## Abstract

The increasing maturity of Internet information technology has led to the rapid rise of blockchain technology. In essence, a blockchain is a shared database. In recent years, blockchain technology has attracted the attention of the public and society. With the continuous development of the market economy, many domestic enterprises have grown in size. At the same time, companies are also faced with various risks, and business risks will have a great impact on the company's production. This article aims to prevent the business risk of Internet information security platform enterprises based on blockchain technology. Through the PoS algorithm, PoW algorithm, secure hash algorithm, and the principle of direct trust, the Internet information security platform is designed. Firstly, the platform is used for a business risk test with a small company, and the platform satisfaction survey is conducted on the employees of the company. The test results show that the subplatform design reduces the business risk of the company by 5%–10%, and employee satisfaction is high. The signature simulation of this algorithm under the same conditions as the SMRA and RSAR methods is also carried out. The results show that the performance of this algorithm is better. This study opens up a new path for small and medium-sized enterprises to prevent business risks.

## 1. Introduction

Due to the complexity of current market issues and fraud, some companies do not understand preventive measures and have little understanding of legal issues in their business, making them unable to effectively avoid operating risks. Blockchain is an important concept of bitcoin. In essence, it is a decentralized database [1]. In a narrow sense, blockchain is a chained data structure that combines data blocks in chronological order, and a distributed ledger that cannot be tampered with and forged in a cryptographic way [2]. Broadly speaking, blockchain technology is a new distributed infrastructure and computing method that uses blockchain data structures to verify and store data, uses distributed node consensus algorithms to generate and update data, uses cryptography to ensure the security of data transmission and access, and uses intelligent contracts composed of automatic script code to program and operate data.

The essence of blockchain technology is a decentralized database, and its main feature is to provide digital trust. Information on the Internet is transparent and anonymous. It is this characteristic that makes information extremely insecure, and information loss, theft, and forgery are very common, which makes the Internet have some information security risks. If this problem cannot be resolved in time, it will seriously affect people's trust in the Internet and drive people away from the Internet. Only by comprehensively preventing the Internet information security platform from corporate management risks can we effectively guarantee Internet information security and reduce corporate operating risks. Improve the company's information risk management capabilities and raise the company's management level to the international advanced level, which provides a strong guarantee for the company's international development and cooperation. This paper aims to propose an effective business prevention scheme for the Internet platform based on blockchain technology to ensure the information security and transaction security of enterprises.

Technical personnel such as Viana E. proposed an Android-based solution for smartphones to identify and report potentially unsafe settings and developed an application that can check smartphones to search for unsafe user configurations based on a predefined list. It reduces the attack of netizens by malicious users [3]. But at that time, they did not use the blockchain technology that has been particularly popular in recent years to reduce the risk of such Internet security information leakage. Researchers such as Bendul J C identified corporate risk culture and product vulnerability as the main factors influencing the implementation of preventive activities during transportation. Regression analysis illustrates the relationship between risk and quality-related influencing factors and the shipper's ability to perform risk prevention activities [4]. But they only studied the corporate risk culture and did not conduct in-depth research on the prevention of corporate operating risks. Scientists such as JJ Sikorski emphasized cryptocurrency mankind's research and practice potential in relation to the 4th industrial revolution. They came to the conclusion that bitcoin has the possibility to be underutilized in addition to supporting and boosting the industrial rebellion's efficiency, and they have defined the subject of future work [5]. However, they did not apply blockchain technology to Internet information security management and risk prevention in business operations. The above research contents are scientific and technological research on risk prevention, which can provide some references and ideas for this research. However, some research schemes do not use cutting-edge blockchain technology or do not protect the core content of enterprise risk. These are the key points of this research.

Protecting the security of information on the Internet, when using traditional information protection mechanisms, is difficult to ensure security. In order to better maintain the security of the network environment, the use of blockchain technology can enhance the protection effect, including user information, transaction activities, electronic communications, infrastructure, etc., which can be protected accordingly. A new blockchain-based Internet information security platform will improve information control capabilities and allow users to safely use online information. The experimental part of this paper not only pays attention to the maturity of technology but also has more humanistic characteristics, referring to the user's satisfaction with the platform.

## 2. Blockchain Security Algorithm

### 2.1. Direct Trust Mechanism

The trust mechanism refers to the various parts of the company's system that constitute and influence the mutual trust relationship and the relationship management mechanism between them. Assuming that the lending decision of lender B is not affected by factors such as income and environment, but only depends on the credibility of the borrower, then, when the credibility is *P*(0 ≤ *P* ≤ 1), the business operation risk rate is P.B. The basis for judging the credibility of the borrower's future performance of the contract is the borrower's credit information, where the information set displayed by the borrower *W* on the platform is *W*={*W*_1_, *W*_2_, *W*_3_,…, *W*_*i*_}. In actual situations, W may deliberately conceal unfavorable information or exaggerate certain pieces of information, and its true information set is *W*′={*W*_1_′, *W*_2_′, *W*_3_′,…, *W*_*i*_′}. However, B can only see the set *W*, so the direct trust expectation made is

(1) $$\begin{array}{c} W=c_{1}U_{1}+c_{2}U_{2}+c_{3}U_{3}+\cdots +c_{m}U_{n}. \end{array}$$

*C*_*i*_ (*i* = 1,2,…) is the expected influence coefficient of each information factor on the credibility obtained by B through subjective judgment. The true value of direct trust is

(2) $$\begin{array}{c} W^{\prime }=c_{1}^{\prime }U_{1}^{\prime }+c_{2}^{\prime }U_{2}^{\prime }+c_{3}^{\prime }U_{3}^{\prime }+\cdots +c_{m}^{\prime }U_{n}^{\prime }. \end{array}$$

From the above two formulas, it can be concluded that the enterprise operating risk rate is

(3) $$\begin{array}{c} P\left(W>W^{\prime }|j=k\right)=\frac{1-\left(\sum_{j=0}^{k}{\left(C_{k}^{j}\right)}^{2}/4^{j}\right)}{2}. \end{array}$$

### 2.2. PoW Algorithm

PoW proves that a certain amount of work has been completed at the end of the work. The PoW algorithm has three main components: the work function proof, the retardation and difficulty values, and how to calculate the work function proof. And then use the PoW algorithm to block the input data. The most difficult part of PoW is the amount of calculation. The work end needs to do some difficult work to get a result, but the verifier can easily check whether the work end has done the corresponding work through the result. The benefits of the PoW algorithm include complete decentralization, free entry and exit of nodes, simple algorithms and simple implementations to reach consensus between nodes without exchanging other information [6, 7]. This algorithm is highly secure and requires a lot of damage to the system funds and allow 50% of the nodes in the entire network to fail. The PoW algorithm also has many shortcomings. For starters, it necessitates a significant amount of computational power, is susceptible to less supervision, and poses security hazards. Simultaneously, the introduction of huge mining tanks has brought attention to the issue of computational capacity, namely the potential of a “51 percent attack.” The performance is low, but whenever a resolution is formed, the entire network is required to join in the computation. Reaching an agreement is impossible, disagreements are prone to occur, and a large number of confirmations must be waited for. The following are the specifications for the structure of chunk *H* said by a node in PoW: *B* is a particular hash technique, where *T* is a set quantity in *H*(*A*)target. That is, the hash value in its entirety. The chunk must be less than the stated amount and include a specific number of locations. The block is a lawful block such that if it fits this criterion, other nodes will accept it. If the node finds such a lawful zone, it will compensate the mines excavated with particular digital money. It also overcomes the problem of several distributed nodes causing problems with judgment. The overall chance *P* of discovering a valid chunk within every test, provided the greatest checksum is *H*, is

(4) $$\begin{array}{c} P=\frac{T_{\text{target}}}{H_{\max}}. \end{array}$$

Clinched alongside Bitcoin, the worth of *t* is balanced each 2016 obstructs (two weeks), which may be balanced toward the taking after formula

(5) $$\begin{array}{c} T_{\left(\text{new}\right)}=\frac{T_{2016}}{2W}\cdot T_{\text{tar}}. \end{array}$$

Around them, *T*_2016_ speaks to the duration of the time expended should produce the past 2016 territory squares. At those duration of the time expended may be shorter, those last focus quality will be Additionally more modest. Those challenge esteem of the created piece might make acquired toward recipe 3:

(6) $$\begin{array}{c} D_{\left(\text{difficulty}\right)}=\frac{T_{1}}{T_{\text{current}}}. \end{array}$$

### 2.3. PoS Algorithm

The PoW (proof of work) is the proof of workload, also known as mining. Most public chains or virtual currencies, such as bitcoin and Ethereum, are based on the PoW algorithm to realize their consensus mechanism. That is, the distribution of money is determined according to the effective work of the mining contribution. Compared with PoW, the PoS algorithm avoids a large amount of waste of resources caused by mining, reduces the consensus time between different nodes in a good low-level network environment, reaches the millisecond level, and has a large number of advantages. A PoS is a method of obtaining accounting rights based on decentralized computing competition. The supervisory ability is weak and has the same fault tolerance as PoW. It can be found in many different PoS applications that this is a hybrid way of using account balance custom mining (where *b* represents the account balance and *t* is a timestamp)

(7) $$\begin{array}{c} H\left(B,t\right)\leq b*T_{\left(\text{target}\right)}. \end{array}$$

### 2.4. Blockchain Data Security Design

Blockchain is an important concept of bitcoin. In essence, it is a decentralized database. At the same time, as the underlying technology of bitcoin, it is a series of data blocks associated with cryptographic methods. Each data block contains a batch of information about bitcoin network transactions, used to verify the validity of its information (anticounterfeiting) and generate the next block. This article aims to improve the security and anonymity of blockchain transactions. For the signing algorithm of blockchain transactions, which cannot resist quantum computing attacks and the security problem of user identity privacy leakage, the research on key technologies for transaction security and privacy protection of blockchain has been carried out. The main research results of this paper are as follows:

Generation of key: randomly select two large prime numbers *p* and *q* to calculate: *n* = *pq*, *Q*(*n*)=(*p* − 1)(*q* − 1), then select either positive integer *e* and calculate *d* so that de = 1 mod *Q*(*n*), where *e* is the public key and *d* is the private key.

The clear text encryption formula for the encryption process is

(8) $$\begin{array}{c} C=M^{e}\mathrm{mod}n. \end{array}$$

The ciphertext decryption formula for the decryption process is

(9) $$\begin{array}{c} M=C^{d}\mathrm{mod}n. \end{array}$$

The user uses the public key set *L* and his private key SK to generate a signature (*r*, *s*) as follows:

(10) $$\begin{array}{c} s=\left({\left(1+SK\right)}^{-1}\left(k-rd\right)\right)\mathrm{mod}n. \end{array}$$

Using the sender node *i* message content and the public key as input to obtain the message verification code using formula (11), we get

(11) $$\begin{array}{c} \text{HMAC}\left(PK_{i},S_{i}\right)=H\left(PK_{i}|S_{i}\right), \end{array}$$

where PK is the public key of *i*, *S* is the message content, and *H* is the hash function. Blockchain users in this distributed network, the signature is verified in the following way, and the miner verifies the transaction through the following two formulas:

(12) $$\begin{array}{c} e\leq 2s\sqrt{m},\;e\neq 0,\\ pk_{a}e=\sum_{i=1}^{d}{\left(-1\right)}^{M\left[i\right]}C_{i}. \end{array}$$

The lattice signature algorithm used in transactions in the quantum blockchain scheme after this chapter satisfies the correctness requirement. The protocol process knows the tail signature *e*=*e*′ − *u*. Thus, the following inequality can be obtained:

(13) $$\begin{array}{c} e\leq e^{\prime }+a\leq 2s\sqrt{m}. \end{array}$$

Since *A*_1_(*e*′ − *a*)=(*A*_1_*e*′ − *A*_1_*a*), we can output

(14) $$\begin{array}{c} e^{\prime }\leftarrow S\text{ample Pre}\left(A_{1},S_{ms},b,s\right). \end{array}$$

The signature satisfies *A*_1_*e*′=*b*. We get

(15) $$\begin{array}{c} A_{1}e=A_{1}\left(e^{\prime }-a\right)\\ =b-A_{1}a\\ =\sum_{i=1}^{d}{\left(-1\right)}^{M\left[i\right]}C_{i}+A_{1}a. \end{array}$$

Through the analysis of equations (13) and (14), it is proved that the lattice signature algorithm used in the proposed postquantum blockchain scheme transaction satisfies the correctness.

ECC (error checking and correction) is error detection and correction algorithm for NAND. For the same key length, the key length of the ECC algorithm grows slowly, while the key length of the RSA algorithm grows exponentially, as shown in Table 1.

## 3. Design and Innovation of Internet Information Security Platform Based on Blockchain Technology

### 3.1. Blockchain Technology to Build a Distributed Model of Internet Information Security Platform

Blockchain technology creates a distributed model for specific applications. The distributed model places the data that different users need to access different parts on different servers to realize horizontal expansion. All users participate in the maintenance of the database. Use encryption technology to create data blocks and interconnect the data blocks [8, 9]. These interconnected data blocks are called blocks, and the data blocks are connected in chronological order to form a blockchain. Each block contains a time period, and the content in the block is the new information generated during the time period, and which covers the anticounterfeiting mark used to verify the information. During the information submission process, the information can only be retained in the database with the approval of the developer and cannot be deleted or changed at will. In terms of architectural design, the architecture of an Internet information security platform based on blockchain technology is shown in Figure 1.

### 3.2. Core Technology of Enterprise Operation Risk Prevention Based on Blockchain

The secure hash algorithm is an encryption technology [10]. It is to transform the input of any length into an output of a fixed length through a hash algorithm, and the output is the hash value. This transformation is a compression mapping; that is, the space of the hash value is usually much smaller than that of the input, and different inputs may be hashed into the same output. In short, it is a function that compresses messages of any length into a message digest of a fixed length. In the data calculation process, if the corresponding hash value is calculated in the forward direction, the calculation process is easy. When the hash value is used, the calculation of the corresponding data is an inverse calculation, and it can be known that this calculation is somewhat difficult. Blockchain networks use hash trees to perform calculations, which are used to construct a Merkle tree whose nodes are hash values. This method can verify the authenticity of a large amount of data. For example, in the security verification process, if a transaction is executed on the double flower subchain, the hacker will find a strong block in the network environment and create a weaker block with a higher cost before that. Judging from the displayed results, if the confirmation time is 1 minute (in 1 MB blocks), a double-spending attack is required. Hackers may occupy 20% of the computing power of the entire network, and the hacking fee will reach 0.8 US dollars. If the block is 4 MB, the double-spending attack will need to pay a high transaction fee of more than $40. This type of security level is relatively low, and its security is similar to that of Bitcoin. Tables 2 and 3 show the transaction security of the security confirmation [11,12].

Analysis of the data in Tables 2 and 3 shows that as the information in the random block changes, its own Merkle hash also changes, and the information contained in the next block also changes. If hackers forge information, their computing power does not support false blocks, and the speed of false blocks exceeds the growth rate of the blockchain and is discarded [13, 14]. The information in each block is not only text information, but also data information, including nonlinear information (such as video information, image information, and various structured messages). The information stored in all blocks will be permanently protected and cannot be maliciously modified. Therefore, blockchain information is relatively safe [15–17].

## 4. Prevention of Business Risks of Internet Information Security Platform Enterprises

### 4.1. Necessity of Building an Internet Information Security Platform

Because this article uses the Fabric blockchain platform, it provides pluggable module configuration and management, by writing-related programs to implement the group signature scheme, and then using the RPC protocol in the blockchain network to remotely call the scheme of this article by controlling the upstream and downstream of the swarm nodes. We verify that our improved scheme can implement dynamic join and exit of nodes, as shown in Table 4.

After designing a blockchain-based Internet information security platform, we applied this platform to a small company to conduct a one-month business risk test. The test results are shown in Figure 2.

It can be seen from Figure 2 that in the first ten days of the year, the Internet information security platform was still in the debugging stage, and information security leaks were more serious. In particular, hackers attacked the system and employee login accounts were stolen. Vulnerability repairs have reduced the probability of various information security incidents by more than half in just over 10 days from early to late. This also proves that the Internet security platform can greatly reduce business risks, and the construction of an Internet information security platform is effective for the company. It is urgent to say [3, 18].

### 4.2. Corporate Employees' Satisfaction Survey on Internet Information Security Platforms

The data structure of blocks in a blockchain-based supply chain management system is shown in Figure 3.

The dotted box in Figure 3 corresponds to the data layer, the categorical Merkel tree layer, the classification Merkel tree root layer, the directory layer, and the block header layer in the block data structure, respectively.

For the supply chain with a production enterprise as the core, the operation process is described according to the order of business operation, so the process of generating the corresponding information for a certain business entity is also carried out according to the supply chain operation business process. The network of virtual links between a business principal's information in a blockchain-based supply chain is shown in Figure 4.

After a one-month risk test, we conducted a questionnaire survey on the company's employees of different age groups on their satisfaction with the platform design. We distributed 110 questionnaires and recovered 110, of which 2 were invalid questionnaires and the rest. There are 108 valid questionnaires in total, and the statistical results are shown in Figure 5.

It can be seen from Figure 5 that more than 50% of employees are very satisfied with the design of this security information platform. They believe that this platform can greatly reduce business risks and increase the company's net income. Less than 10% of employees are dissatisfied with the platform and think. This platform still has a lot of shortcomings, such as the design page is too simple, the system functions are not rich enough, etc.

### 4.3. Confidentiality Measures for Blockchain Electronic Signatures

For ring signatures, it has the following characteristics: *Correctness.* If the user can sign the signed message according to the correct signing steps and it has not been tampered with, then during the verification phase, the resulting ring signature must meet the ring signature verification formula. *Unconditional anonymity.* It is almost impossible to determine the true identity of the signer. Assuming that there are *n* members participating in the ring signature, even if the attacker steals the private keys of all voters by some means, the chances of him being able to successfully identify the true signer of a signature will be less than 1/*n*. *Unforgotten.* It is difficult to successfully forge a legitimate signature. In the whole process of ring signing, the verification process of each ring member is different, and the signature result is the same. In this case, it is difficult to counterfeit.

Blockchain technology is a decentralized distributed database technology with the characteristics of trustlessness, transparent transaction openness, and immutable data, which can effectively reduce data management costs, improve work efficiency, and protect data security. However, with the development of quantum computing, quantum computing attacks with strong computing power can crack classical cryptographic algorithms, which poses a huge threat to transaction security that relies on elliptic curve digital signature algorithms to ensure the transaction security of the blockchain. At the same time, due to the transparency of transaction information on the blockchain, relevant research has proved that there is also a risk of user identity privacy leakage [19]. Therefore, research on blockchain transaction security and privacy protection has become an important topic in the current blockchain security field.

Since the concept of electronic voting was first proposed in 1981, its basic model can be summarized as shown in Figure 6.

This paper designs an experiment to compare and analyze the signature generation times of the SMRA algorithm and the RSA-based signature algorithm RSAS, and the experimental data is shown in Table 5.

The above data shows that in the case of an equal number of ring members, the signature generation time of the SMRA algorithm is less than that of the RSAS algorithm, and the signature efficiency is higher. Based on the above data, this article draws a simulation diagram as shown in Figure 7.

Through simulation experiments, the performance efficiency of the protocols is compared. The public key length, private key length, and signature length of the scheme in this section and the SMRA and RSAS methods are tested respectively, and *q* = 2^10^, *d* = 64, and *m* = 6*n*log*q* are set under reasonable parameters according to the actual requirements in the lattice cryptographic algorithm, we set the security parameter *n* range from 10 to 160 increments, in turn, 16 tests. The experimental test results of public key length, private key length, and signature length for each scenario are shown in Figures 8–10, respectively.

Simulation test results show that with the continuous increase of the security parameter *n*, the public key, private key, and signature length of this section scheme are shorter than other schemes. In summary, the proposed signature algorithm has a relatively short one.

## 5. Conclusion

Internet information security issues are diverse, which means that Internet companies and users should have a sense of prevention when using the Internet and actively use new technologies to build an information security fortress on the Internet so as to reduce business risks. The development of blockchain technology provides a new model for Internet information security that is completely different from traditional forms of security prevention. The use of blockchain to develop Internet information security platforms can effectively protect the information security of enterprises. For example, a user's basic information, transaction information, and contact information can be guaranteed, thus greatly reducing the risks of business operations. But it should also be pointed out that any technology is a double-edged sword, with opportunities and challenges. The development of new technologies inevitably faces risks, and the blockchain is the same. Therefore, in the process of applying blockchain technology, we should think carefully, study carefully, make full use of the benefits of blockchain technology, and create an excellent new information security platform on the Internet that contributes to the prevention of business risks.

## Figures and Tables

**Figure 1:** Internet information security platform based on blockchain technology.

**Figure 2:** Business risk test.

**Figure 3:** Data structure of blocks in a blockchain-based supply chain management system.

**Figure 4:** Blockchain-based virtual link network of information of a business entity in the supply chain.

**Figure 5:** Enterprise employee satisfaction survey.

**Figure 6:** Diagram of the basic model of electronic voting.

**Figure 7:** Simulation result graph.

**Figure 8:** Public key length comparison result.

**Figure 9:** The result of the private key length comparison.

**Figure 10:** Signature length comparison result.

**Table 1:** Comparison of ECC and RSA key lengths.

Symmetric key length (bit)	RSA key length (bit)	ECC key length (bit)
86	1024	32
68	2048	16
16	3074	64
64	7660	4
54	14230	256

**Table 2:** 5 seconds to confirm the security of the transaction after being confirmed in the double flower subchain.

The hash power of bad intruders is the mutual percentage in the network (%)	The estimated cost of a successful double-spending supply confirmed in 5 seconds (*μ*B)		
	1.0 MB block	2.0 MB block	Probability of success (%)
0.05	600	1200	10
0.15	210	420	23.2
1.32	40	80	52.6
2.52	30	60	76.2
15	15	30	92.3
20	5	10	95.6

**Table 3:** 10 seconds to confirm the security of the transaction after being confirmed in the double flower subchain.

The hash power of bad intruders is the mutual percentage in the network (%)	The estimated cost of a successful double-spending supply confirmed in 10 seconds (*μ*B)		
	2.5 MB block	5.0 MB block	Probability of success (%)
0.08	1500	3000	20
0.23	210	420	33.2
1.35	80	160	66.2
2.80	60	120	79.2
18.2	20	40	95.1
24.6	10	20	98.5

**Table 4:** Experimental environment configuration.

Configuration item	Configuration parameter
Operating system	Ubuntu 16.04 64 bit
CPU	Intel ® Xeon ® Platinum 8269CY 2.5 GHz
RAM	4G
Maximum network bandwidth	200 Mbps

**Table 5:** SMRA and RSAS signature time comparison analysis.

Number of ring members SMRA	Signature generation time (ms)	RSAS signature generation time (ms)
1	16.54	21.57
5	17.92	23.54
10	19.72	25.03
20	20.81	26.9
50	22.72	28.79
80	24.03	30.34
100	25.9	31.46
150	27.35	33.2
200	28.51	35.06
300	30.39	36.37

## Data Availability

No data were used to support this study.
